The article "Temporal and Spatial Differences of Urban Ecological Environment and Economic Development Based on Graph Neural Network" was retracted in 2023. Reasons: signs of a paper mill; suspected computer-generated content; unreliable results or conclusions; concerns about the data.

# Temporal and Spatial Differences of Urban Ecological Environment and Economic Development Based on Graph Neural Network

**DOI:** 10.1155/2022/7078671

**Published:** 2022-06-21

**Authors:** Wenbo Zhang, Binggeng Xie

**Affiliations:** ^1^College of Resources and Environmental Sciences, Hunan Normal University, Changsha 410081, Hunan, China; ^2^School of Geography and Environmental Engineering, Gannan Normal University, Gannan 341000, Jiangxi, China

## Abstract

The temporal and spatial difference between the urban ecological environment and economic development refers to the unbalanced and insufficient contradiction between the quality of urban ecological environment and the development of economic strength. Based on the relevant theories of urban ecological environment and economic development, this paper explores the development laws of urban ecology and economic development and uses graph neural network algorithm to model the spatial and temporal dependence of the city's ecological environment in a province. The quality data and economic development strength data are analyzed in detail. The analysis results show that the ecological benefit index and economic benefit index of each city in the province have reached above 0.6 after 5 years of development. The level of coordinated urban development has improved significantly compared with 2017. However, in the process of the development of the market economy, it is necessary to rationally adjust the proportion of the secondary industry and the tertiary industry in the urban production structure and continuously promote the balanced development of the economy and ecology.

## 1. Introduction

Since ancient times, how to find a balance between the ecological environment and economic development has always been an important issue in the process of human development. With the improvement of human society and the level of the times, the market economy has achieved unprecedented in-depth development. A strong economic foundation can provide greater support for the construction of green and harmonious ecological environment, but the market has always focused on economic development, while ignoring the construction of the ecological environment. To a certain extent, this has resulted in the spatial and temporal differences between the urban ecological environment and economic development. This temporal and spatial difference not only causes the serious problem of ecological environment deterioration but also hinders the sustainable development of social economy. As shown in Figure 1, under such a severe situation, the research on promoting the harmonious development of the ecological environment and economy has become the focus of attention from all walks of life. Since the second half of the 20th century, in order to promote the balance of economic and ecological structures among various urban areas, a large number of scholars have conducted investigations and studies on this. However, the research form is single, and many research results are only for individual cities and regions and are not representative.

With the rapid development and continuous improvement of science and technology, the application of machine learning algorithms in many important value fields has become more and more extensive, such as data mining, medical diagnosis and treatment, finance, computer vision, and natural language processing, and other industries have played its high application value. As one of the important components of machine learning algorithms, neural network models formed by deep learning methods have also demonstrated their excellent performance in various industries. Especially when people need to perform scene analysis to make important decisions in their daily life, the value of neural network models is particularly important. Each node of the graph neural network model has close associations, and this association hides very important structural information, and the graph neural network algorithm can give full play to the existing value of this structural information. It needs to continuously analyze, process, and dig out more content information data to assist decision-making. It can quickly analyze the important factors affecting decision-making while ensuring the accuracy of decision-making and provide a credible decision-making basis, so as to better serve people's lives. On the whole, due to the special superior performance of graph neural network, it is often used for relational reasoning and information integration of scenes, which has certain academic and social value.

In recent years, many scholars have carried out research on technique of algorithmic graph neural networks. Aiming toward the limitations of existing graph neural networks, Na *G* S et al. comprehensively analyze the structure of graph neural networks and develop a cost-free molecular analysis solution for the limitations of graph neural networks. Finally, they verified the usefulness as a solution by conducting experimentation with a variety of reference sets of data [1]. Lee L H. et al. proposed a graph neural network model for medical applications. They integrate several implementations at distinct particle sizes from root, string, and word levels into the neural network of various governor diagram series and finally validate the operability of the model with an experimental dataset [2]. N Guo et al. proposed a graphical nerve nets' algorithm-based SOC estimation model, which has been improved through a combination of graphical nerve nets and amperometric integration. Finally, a simulation test was carried out to verify the superiority of the algorithm [3]. Scalia *G* et al. compare scalable techniques for imprecision detection within graphical involutional nerve grids, quantifying the behavior of various imprecision determination schemes as well as their influence on inequality-related mistake mitigation. Such techniques contribute to a greater awareness of the effects of contingent indeterminism on certainty [4]. Li Z et al. suggested a discriminative dictionary learning algorithm based on graph neural network; they classified images based on the best coding coefficients obtained from local and label reconstruction. Laboratory findings indicate that the technique can perform significantly faster compared to a number of cutting-edge techniques [5]. Qi Y et al. present a mixed computer system with a deep learning methodology. The model combines a graph deconvolutional network as well as a gap linear short-term memory network to simulate and forecast the quantitative changes in PM 2.5 concentration in space and time, and according to the results, the model has the best performance in prediction [6, 7]. Luo Z et al. proposed a convergent nerve grid model using Ngram-based patches for graph recognition. They verified the effectiveness of the method by making a benchmark against available state-of-the-art measures with five authentic galleries of maps coming from various fields of bioinformatics and public networks [8]. Zhang Y M et al. propose an efficient and robust graph-based method for transduction classification for public datasets and web spam detection. The detection experiment proves that this approach provides the benefit of high accuracy and rapidity [9]. Geyer F et al. proposed a performance prediction method based on graph-gated neural network. They used this method to predict the throughput of TCP flows and the delay task of UDP flows and verified its effectiveness [10]. Yan H et al. proposed a graph neural network multiview method for acquiring several midlevel functions for better verification performance. Finally, they demonstrate the excellent validation ability of the proposed method on four publicly available experimental datasets [11]. In summary, after several years of exploration, the application of graph neural network algorithm technology has been deeply studied by many scholars, but there are not many studies that integrate it with the spatial and temporal differences of urban ecological environment and economic development. Therefore, in order to further facilitate a balanced growth of the urban ecosystem and society, it is urgent to study the temporal and spatial difference analysis of urban ecology and economy from the perspective of graph neural network algorithm technology.

Based on the graph neural network algorithm technology, this paper proposes a novel research direction on the spatial and temporal differences between urban ecological environment and economic development. This technology can effectively make accurate judgments on the temporal and spatial differences between urban ecological environment and economic development, provide suggestions for improvement and improvement of urban development under machine learning algorithm technology, and provide new ideas for the research of urban development.

## 2. Related Work

Theory of man-land relationship: for a long time, the theory of human-land relationship has been a hotly discussed issue in geography. Human-land relationship refers to the interaction and interaction between humans and the geographical environment. It not only includes the natural understanding and natural creation of the geographical environment by human beings in the process of evolution and activities but also includes the role and impact of natural understanding and natural creation on the geographical environment, and the role and influence here are dual, both positive and negative. With the continuous acceleration of the development process of human society, human beings' natural understanding and natural creation of the geographical environment are also constantly changing and adjusting. The understanding of human-earth interaction and mutual influence is also deepening, and this depth has diversity and historical differences. Diversity refers to the diversity in the definition of the human-land relationship, which is reflected in two levels of individuals and perspectives. From an individual point of view, most scholars will conceptualize the human-land relationship based on their own research. Although they are generally the same, they are different in subtleties. Nowadays, there are many different man-earth views in geography, including environmental determinism, cultural determinism, destiny theory, and adaptation theory; from an angle, the concept of the man-earth relationship can be defined from a narrow perspective and a broad perspective.

The development and progress of the times not only promote the rapid improvement of the social and economic level but also promote human beings' cognition of the relationship between man and earth. As a result, to correctly find a balance between the ecological environment and economic development, the way of thinking and practical activities of human beings are constantly being adjusted. From blindly focusing on and pursuing social and economic development to the serious imbalance and deterioration of the urban ecological environment, human beings have shifted the urban ecological environment to the focus of development. And then apply the concept of shared destiny to the solution of the problem of spatial and temporal differences between urban ecological environment and economic development. However, no matter what measures are taken, they should be based on the premise of reverence for nature and respect for the laws of nature, rationally exert the application value of the geographical environment, continuously reduce the negative impact of economic activities on the ecological environment, and strive to achieve a shared destiny and harmonious coexistence of man and nature.

Environmental economics theory: environmental economics theory is developed on the basis of economics theory, mainly from the perspective of economics theory. Social science applies the analytical methods of economics to deeply study the principles of interaction between the urban ecological environment and the economy. Since the second half of the 20th century, the world industrial revolution has not only brought about a rapid rise in the level of global economic development but also brought about the destruction of the ecological environment, and thus, the theory of environmental economics was born. And with the continuous improvement and development of the times, the research field of disciplinary theory is also continuously expanded, and the research content has changed from a single perspective to a variety of perspectives. It not only analyzes the principle of mutual influence and interaction between urban ecological environment and economy but also analyzes and studies the role and means of environmental protection and the sustainable development of economy. The practice of human beings to really deal with the urban ecological environment begins in production because it is well known that the destruction of the urban ecological environment is mostly caused by production activities. Therefore, the theory of environmental economics studies the core issues of the urban ecological environment from the perspective of economic analysis and deals with the protection and management of the urban ecological environment by dealing with economic methods and means. This not only provides an economic perspective for the study of the temporal and spatial differences of urban ecological environment and economic development but also pays attention to the value cost of environmental management.

Sustainable development theory: the concept of sustainable development was proposed in 1987. The World Commission on Environmental Development (WCED) submitted a very important and valuable research report to the United Nations based on the concept of the harmonious development of ecological environment and economy, which mentioned sustainable development. This concept has received strong attention from countries all over the world because countries all over the world are facing the question of whether social development is sustainable. The concept of sustainable development in the research report is a comprehensive strategy, which faces the entire human society and aims to solve the temporal and spatial differences between urban ecological environment and economic development, find a balance point, and maintain a harmonious and symbiotic development state. In the course of development in the new century, people are constantly aware of the importance of the ecological environment, so it is particularly important to analyze and resolve the temporal and spatial differences between urban ecological environment and economic development with the concept of sustainable development as a development strategy.

Ecological economics theory: ecological economics theory is different from environmental economics theory. Ecological economics refers to the discipline that combines ecology and economics to study the structure, function, and movement law of the complex system of the ecological system and economic system, which is a discipline that studies the system structure of the ecological economy and explores the laws and principles of system development.

Human society mainly relies on the production of labor to promote progress and development, and the relationship between human society and the ecological environment has mainly gone through three stages, which are the agricultural society stage, the industrial society stage, and the ecological economy stage. In the stage of industrial society, the development contradiction between human society and the ecological environment is particularly obvious. It was also at this stage that scholars began to realize that the temporal and spatial differences between urban ecological environment and economic development could not be alleviated at all from a single perspective of ecology or economics because, at this stage, the environmental problems and pressures brought about by industrial production have reached a point that cannot be ignored. In the long run, human society will usher in a seriously unbalanced living environment, but even economic development will be greatly hindered. Only by combining economics and ecology with each other, it is possible to find the law of development and alleviate the development contradiction. The theory of ecological economics analyzes the dynamic laws of the ecological economic system from the perspective of ecology and economy. It believes that all production activities of human society are carried out in the ecological economic system. When coordinating the interaction between the urban ecological environment and economic development, it needs to consider not only the natural development law of the ecological environment but also the economic development law. Therefore, on the basis of the theory of ecological economics, the relationship between the two is coordinated from the ecological economic system, to find a dynamic balance and redistribute to play their respective application values. It is applied in protection and reasonably solves the temporal and spatial difference between urban ecological environment and economic development in the development process of production practice.

## 3. Graph Neural Network Model

### 3.1. Definition of Diagram

A graph is a commonly used data structure, which generally consists of a set of vertices and a set of edges between vertices. Among them, the vertex can be a research object, and the edge corresponds to the relationship between different research objects. The graph can usually be expressed as. The meaning of each parameter is shown in Table 1.

The set of connected edges in Figure *G* can be represented as *E*={*e*_1_, *e*_2_,…, *e*_*m*_}, where *m* represents the number of connected edges in the graph. In addition, the connecting edge between vertex *V*_*i*_ and vertex *V*_*j*_ can be represented as *e*_*ij*_. If the connected edges in the graph have no direction, the graph at this time is an undirected graph, so there is [12]

(1) $$\begin{array}{c} e_{ij}=e_{ji}. \end{array}$$

There are various storage representations for graphs, such as adjacency matrices and adjacency lists. As shown in Figure 2, the adjacency matrix is the most widely used and easy to combine with matrix operations.

Adjacency matrix *A* ∈ *R*^*n*×*n*^ is defined as the following formula:

(2) $$\begin{array}{c} A_{ij}=\left\{\begin{array}{cc} 1 & e_{ij}\in E,\\ 0 & \text{otherwise}. \end{array}\right.. \end{array}$$

That is, when there is an edge *e*_*ij*_ between vertex i and vertex *j*, the element corresponding to *A*_*ij*_ is 1, otherwise it is 0.

The degree matrix of a graph is a diagonal matrix of degrees of vertices. The elements on the diagonal are the degrees of the corresponding vertices, that is [13–15],

(3) $$\begin{array}{c} D_{ij}=\sum^{}jA_{ij}. \end{array}$$

The Laplace matrix of a graph is an important operator in spectral graph analysis, and its structure is shown in Figure 3.where *I*_*N*_, *A*, and *D* represent the identity matrix, the adjacency matrix, and the degree matrix of the graph, respectively.


(4) $$\begin{array}{c} L=I_{N}-D^{-1/2}{\;}^{*}A{\;}^{*}D^{-1/2}, \end{array}$$

(5) $$\begin{array}{c} L=D^{-1/2}{\;}^{*}\left(D-A\right){\;}^{*}D^{-1/2}. \end{array}$$

Since the Laplacian matrix *L* is a real symmetric matrix, the Laplacian matrix *L* can be further decomposed as follows:

(6) $$\begin{array}{c} L=U\Lambda U^{T}, \end{array}$$

where *U* represents the matrix formed by the eigenvectors of the Laplacian matrix, and the elements on the diagonal of Λ represent the eigenvalues of the Laplacian matrix.

### 3.2. Calculation of Graph Convolution

Unlike traditional convolutions that are often used in fields such as image processing and computer vision, graph convolutions are often used to perform convolution calculations on graphs, as shown in Figure 4.

Specifically, graph convolution can be defined as the operation between signal *x* and filter *g*_*θ*_ in Figure 4, as shown in the following formula [16]:

(7) $$\begin{array}{c} g_{\theta }*g^{x}=g_{\theta }\left(L\right)x=g_{\theta }\left(U\Lambda U^{T}\right)x=Ug_{\theta }\left(\Lambda \right)U^{T}x,\\ g_{\theta }*g^{x}=Ug_{\theta }\left(\Lambda \right)U^{T}x, \end{array}$$

where *∗g* represents the graph convolution calculation.

However, computing the multiplication between multiple different matrices is very time-consuming. Since *g*_*θ*_(Λ) is a diagonal matrix, the time complexity here is only *O*(*n*^2^). Furthermore, computing the eigendecomposition of Laplacian matrix, *L* also takes a lot of time. These situations are exacerbated when faced with large-scale graphs.

In order to further reduce the computational complexity and enable the filter to be localized, the filter function *g*_*θ*_ can be approximated by a *k*-order Chebyshev polynomial. Among them, the recursive form of the Chebyshev polynomial is shown in the following formula [17]:

(8) $$\begin{array}{c} T_{k}\left(x\right)=2xT_{k-1}\left(x\right)-T_{k-2}\left(x\right), \end{array}$$

(9) $$\begin{array}{c} T_{0}\left(x\right)=1, \end{array}$$

The improved graph convolution computation based on Chebyshev polynomial approximation can be defined as follows:

(10) $$\begin{array}{c} g_{\theta }*g^{x}=\sum_{k=0}^{K}\theta_{k}T_{k}\left(\tilde{L}\right)x, \end{array}$$

(11) $$\begin{array}{c} \tilde{L}=\frac{2}{\lambda_{\max}}L-I_{N}, \end{array}$$

where λ_max_*x* is the largest eigenvalue of Laplacian matrix *L*.

As shown in Figure 5, when *K*=0, the graph convolution only considers the input features of its own nodes and updates its own feature representation during calculation. When *K* is equal to 1, the graph convolution will consider not only the input features of each node but also the input features of the first-order neighbor nodes of each node when updating the features of each node.

In this paper, we define a graph convolutional layer as follows:

(12) $$\begin{array}{c} x_{l+1}=\text{GCN}\left(x_{l}\right)=g_{\theta }*g^{x}, \end{array}$$

where *x*_*l*_ and *x*_*l*+1_ represent the input features and output results of the *l*th graph convolution layer, respectively.

### 3.3. Diagram Construction

This paper first constructs a relationship graph for all regions of the city to model the complex spatial relationship between different regions. In order to be able to perceive the changes of the whole ecological environment from these adjacent regions and functionally similar regions, this paper proposes a method for constructing a relationship graph, which considers the proximity relationship between different regions.

According to the first law of geography, all things are related to other things, but things that are near are more related than things that are far away. Therefore, this paper first considers the spatial relationship between things with similar distances, that is, the proximity relationship. Based on the proximity relationship of regions, this paper determines whether there is an edge between two regions (nodes) according to whether the two regions are in contact with each other. As shown in Figure 6, given a 3 × 3 grid graph, the middle grid will only generate edges with the surrounding 8 grids. Based on this, the adjacency matrix *A*_adj_ corresponding to the adjacent relationship can be obtained.

### 3.4. Fusion of Multiple Relationships

Finally, the adjacency matrix corresponding to the relation graph constructed based on the adjacency relation is defined as follows:

(13) $$\begin{array}{c} A_{\text{comb}}=A_{\text{adj}}{}^{\circ}A_{\text{sim},\theta_{1}}+\left(1-A_{\text{adj}}\right){}^{\circ}A_{\text{sim},\theta_{2}}, \end{array}$$

where “°” represents matrix multiplication by bitwise operation. In formula (13), the interpretation of each parameter is shown in Table 2.

In Table 2, *A*_comb_ indicates the truly relevant regions in the adjacent regions and (1 − *A*_adj_)°*A*_sim,*θ*_2__ indicates the more relevant regions in the nonadjacent regions. Considering that the degree of proximity between different regions is different, the relative difficulty should also be different, so we use different thresholds *θ*_1_ and *θ*_2_ to constrain different parts of formula (13).

### 3.5. Modeling of Spatiotemporal Dependencies

In the process of spatiotemporal modeling, spatial context information plays a very important role. In this paper, we propose a spatial context-based long-short-term memory network modeling method SC-LSTM to better utilize spatial context information while modeling temporal dependencies. When modeling temporal dependencies, the proposed SC-LSTM not only utilizes the original city information but also utilizes the extracted spatial context information. The spatiotemporal prediction models proposed by some research studies all adopt the strategy of time series modeling (“modeling time dependency first-then modeling spatial dependency” or “modeling spatial dependency first-then modeling time dependency”) to model the spatial dependence and the time series dependence. Taking “time-dependent modeling first-spatial-dependent modeling” as an example, since time-dependent modeling has no spatial awareness in general, when the time-dependent modeling of the preorder outputs the results, the spatiotemporal distribution of the entire data will change. Different from the relationship between the original input features of each region, the next spatial dependency modeling module will face the changed relationship between the features of each region. This makes the entire spatiotemporal modeling process based on time-series modeling strategy more difficult. The ST-LSTM proposed in this paper enables each region to have a certain spatial awareness when modeling temporal dependencies, thereby alleviating the above problems.

Suppose that, at time *t*, we can obtain the traffic flow matrix *X*_*t*_ ∈ *R*^|*v*|×*p*^ corresponding to the entire city area, where |*v*|=*i* × *j* represents the number of districts in the whole city.

First, we design a spatial context information extraction module. This module mainly includes two graph convolution layers to extract the local spatial context information of each region at each moment, as shown in formulas (14) and (15):

(14) $$\begin{array}{c} m_{t}=\delta \left(\text{GCN}\left(X_{t}\right)\right)\in R^{\left|v\right|\times h_{1}}, \end{array}$$

(15) $$\begin{array}{c} {\tilde{X}}_{t}=\text{GCN}\left(m_{t}\right)\in R^{\left|v\right|\times p}, \end{array}$$

where *δ* is a restricted linear unit. The *p*-dimensional input features of each region are first mapped to a *h*_1_-dimensional vector and then reduced to a *p*-dimensional vector. The spatial context information extraction module here can be regarded as acting as “information encoding-decoding.” Ultimately, the extracted spatial context information can carry important information from relevant regions, such as the characteristics of ecological environment changes in other regions.

Next, the extracted spatial context information is merged with the original urban environment matrix to obtain the input features of the entire time-dependent modeling module, as shown in the following formula:

(16) $$\begin{array}{c} {\hat{X}}_{t}=\left[X_{t},{\hat{X}}_{t}\right]\in R^{\left|v\right|\times 2p}, \end{array}$$

where the *p*-dimension of the input features of the time-dependent modeling module is increased from the original dimension to 2*p*-dimension.

Finally, as shown in formula (17), this paper uses a shared layer across all regions of the city to model temporal dependencies. The used layer is used to learn an implicit feature vector from the time series composed of environmental features and context information of each region, so as to mine the time series features in the historical time series of each region:

(17) $$\begin{array}{c} {\hat{H}}_{t-1}^{i}=\text{LSTM}\left({\hat{X}}_{t-T}^{i},\cdots ,{\hat{X}}_{t-2}^{i},{\hat{X}}_{t-1}^{i}\right). \end{array}$$

Modeling spatial dependencies: the temporal features learned by temporal dependency modeling will be directly used for spatial dependency modeling. Specifically, the latent feature vector learned by each region after SC − LSTM will be directly used as the input feature of spatial dependency modeling. When modeling spatial dependencies, we continue to use graph convolution to learn more new features from the spatial dimension. The designed spatial dependence modeling module is defined as the following formula:

(18) $$\begin{array}{c} X_{\text{res}}=\sigma \left(g\left({\hat{H}}_{t-1}\right)\right)\in R^{\left|v\right|\times p}, \end{array}$$

where *σ* refers to the tanh function, *g* is the spatial dependence modeling function, and *X*_res_ refers to the urban area ecological environment matrix predicted by the ecological environment matrix at the historical moment of the city without using other external features. In this paper, the spatial dependence modeling function consists of several graph convolutional layers. The output of the middle graph convolutional layer will apply ReLU as the activation function to avoid overfitting of the model.

## 4. Spatial and Temporal Difference Analysis of Urban Ecological Environment and Economic Development

This paper firstly trains and optimizes the proposed algorithm on different datasets and then applies it to the analysis of spatiotemporal differences in the ecological environment and economic development of cities in a certain province. In this paper, each dataset is proportionally divided into three parts, as shown in Table 3.

In this paper, the data of the training set are used to train the graph neural network model, the loss function is designed as a cross-entropy loss function, and the Adam optimizer is used to optimize the loss function to learn the network parameters. When the model loss converges, the training of the model is stopped, and for the prediction results of the graph neural network model, the interpretability method is used to explain the prediction results. All interpretation methods are evaluated on the nodes of the test set. The dataset information is shown in Table 4.

The experimental object of the spatial and temporal difference analysis of ecological environment and economic development in this paper is a relatively developed province in the southeast, herein after referred to as *J* province. As of 2021, the total resident population of the five cities in *J* province (city A, city B, city C, city *D*, and city E) has reached 24 million, and the regional GDP has exceeded 4 trillion, an increase of about 8% over last year. The ecological environment bulletin shows that the overall evaluation level of the ecological environment in the province is good. In this paper, the graph neural network algorithm is used to analyze the spatial and temporal differences of local economic development and ecological environment from 2017 to 2021. These include ecological environment quality analysis and economic development strength analysis. The analysis results are shown in Figures 7to 10.

### 4.1. Analysis of Ecological Environment Quality

The urban ecological environment quality analysis mainly uses the graph neural network algorithm to analyze the ecological benefit index, pollution control index, per capita green area, and green coverage rate of each city in *J* province, as shown in Figure 7 and 8:

Figure 7(a) shows the changes in the ecological benefit index from 2017 to 2021. Figure 7(b) shows the change of pollution control index from 2017 to 2021.

It can be seen from Figure 7 that the ecological benefit index of each city in *J* province has increased during the development from 2017 to 2021. Province *J* is a coastal city in the southeast and has always attached great importance to the construction of social and ecological civilization. In 2017, the ecological benefit indices of C and *D* cities were both below 0.5, while in 2021, the ecological benefit indices of all cities in *J* province were all above 0.6, indicating that the province's urban ecological civilization construction has achieved significant results. The reason why the pollution control index of *J* province did not increase as much as the ecological benefit index is that, before 2017, *J* province began to focus on the control of industrial pollution caused by manufacturing in various cities, and the pollution control level of most cities itself is relatively high, so the range of change is small, but we can still see that the pollution control of cities in *J* province has always achieved considerable results.

Figure 8(a) shows the change in green space per capita from 2017 to 2021. Figure 8(b) shows the changes in green coverage from 2017 to 2021.

It can be seen from Figure 8 that the greening construction of cities in *J* Province has been advancing, and the per capita green space area and urban green coverage rate in 2017 have both improved compared with the data in 2021. And in 2021, the green coverage rate of the five cities will reach more than 30%, which means that the green coverage rate of the cities in *J* province has reached the national data requirements for the definition of garden cities. The per capita green area of city *E* is 30.02%, and the green coverage rate is 35.42%, far exceeding other cities. The per capita green space in city B and city C has changed from less than 10 square meters to more than 18 square meters per capita, which is a very obvious progress and improvement in urban greening work.

### 4.2. Analysis of Economic Development Strength

The analysis of urban economic development strength mainly uses the graph neural network algorithm to analyze the economic benefit index, economic strength index, and the GDP proportion of the secondary industry and the tertiary industry in each city in *J* province, as shown in Figure 9 and 10.

Figure 9(a) shows the changes in the economic benefit index from 2017 to 2021. Figure 9(b) shows the changes in the economic strength index from 2017 to 2021.

As can be seen from Figure 9, from 2017 to 2021, the economic benefit index of each city in *J* province has an obvious upward trend. The economic benefit index of city B in 2017 is obviously behind the other four cities, but after five years of continuous urban economic growth. The development has surpassed the economic benefit index of city A and city *D*, with a large increase. In general, the economic benefit index of each city is above 0.6, and the economic development trend is relatively good. Among the changes in the economic strength index of each city, city *E* is far ahead of other cities, which shows that the living standard of residents in this city is relatively high. The economic strength index of other cities also increased due to the increase in the GDP and government revenue of *J* province.

Figure 10(a) shows the GDP proportions of the secondary and tertiary industries in each city in 2017. Figure 10(a) shows the GDP proportions of the secondary and tertiary industries in each city in 2021.

It can be seen from Figure 10 that, from 2017 to 2021, the proportion of the tertiary industry in all cities in *J* province has increased to a certain extent, which is the result of the transformation and upgrading of the industrial structure under the market economy. In 2021, city C even completed the development task of the proportion of the tertiary industry surpassing that of the secondary industry. However, from the data provided by the graph neural network, we can see that there are still a few cities whose economic structure is dominated by the development of the secondary industry. The difference in the proportion of the two major industries in city B in 2017 is 30%, and the difference in the proportion of the industry in 2021 is 16%. Although there has been a significant improvement, the focus of urban development should still be placed on the tertiary industry. At this stage, only by improving the development speed and quality of the tertiary industry can the city's economy achieve the goal of sustainable development.

## 5. Conclusion

Urban development is often hindered by the imbalance between ecological environment and economic level. In order to achieve sustainable social development, the development concept must be based on the harmonious coexistence of urban ecological environment and economic development. This paper analyzes the urban development based on the graph neural network algorithm and provides a scientific basis and decision-making for the future development of the city by measuring the quality of the urban ecological environment and the power of economic development has a guiding role. It is believed that, with the progress and maturity of science and technology, the research on the analysis and solution of the problems of urban ecological environment and the spatial and temporal differences of economic development will develop with higher quality and higher level. Although this paper uses the graph neural network algorithm to conduct in-depth research on the spatial and temporal differences between urban ecological environment and economic development, there are still many shortcomings. My academic level and research ability are limited. In our future work, we will continue to conduct better and more mature analysis and research on the development of urban ecological environment and economy based on existing technologies and means.

## Figures and Tables

**Figure 1:** Illustration of ecological destruction.

**Figure 2:** Adjacency matrix and adjacency list diagram.

**Figure 3:** Schematic diagram of Laplace matrix.

**Figure 4:** Diagram of graph convolution.

**Figure 5:** Schematic diagram of graph convolution calculation.

**Figure 6:** Schematic diagram of creating edges between different regions based on proximity.

**Figure 7:** Analysis of urban ecological benefit index and pollution control index.

**Figure 8:** Urban per capita green area and green coverage rate analysis.

**Figure 9:** Analysis of city economic benefit index and economic strength index.

**Figure 10:** Analysis of the GDP proportion of urban secondary industry and tertiary industry.

**Table 1:** Interpretation of each parameter.

Sequence	Parameter	Paraphrase
1	*G*	A graph
2	*V*={*V*_1_, *V*_2_,…, *V*_*n*_}	Set of vertices in a graph
3	*V*_*i*_	*i*th vertex
4	*n*	The number of nodes in the graph

**Table 2:** Interpretation of each parameter in the formula.

Sequence	Parameter	Paraphrase
1	*A*_adj_°*A*_sim,*θ*_1__	Really relevant areas inthe neighborhood
2	(1 − *A*_adj_)°*A*_sim,*θ*_2__	The more relevant regionsof the nonadjacent regions
3	*θ*_1_	Threshold
4	*θ*_2_	Threshold

**Table 3:** Dataset composition information.

Sequence	Dataset components	Proportion
1	Training set	50
2	Validation set	20
3	Test set	30

**Table 4:** Dataset information.

Dataset	Number of categories	Number of nodes	Number of edges	Number of features
Cora	7	2708	10552	1426
Citeseer	6	3321	9237	3491
Pubmed	3	19717	44173	499
Musae-*F*	4	22470	342008	4364
Musae-*G*	2	37700	573007	4065
Amazon-C	4	13752	561442	752

## Data Availability

The data used to support the findings of this study are available from the corresponding author upon request.
